The article "Intelligent Face Recognition System Based on Universal Design Concept" was retracted in 2023. Reasons: signs of a paper mill; suspected computer-generated content; unreliable results or conclusions; concerns about the data.

# Intelligent Face Recognition System Based on Universal Design Concept

**DOI:** 10.1155/2022/8633846

**Published:** 2022-07-14

**Authors:** Zhijie Li, Kibong Shin

**Affiliations:** Department of Design, Silla University, Busan 46958, Republic of Korea

## Abstract

The rapid development of science and technology, i.e., integrated modules that are actuators and sensors, promotes the comprehensive popularization of intelligent products in people's life. More particularly, with the advent of the hybrid of the Internet of things and artificial intelligence, more and more activities preferably linked to the human beings have been automated and developed. Among those fields, intelligent face recognition has also become a basic technology in work and life. This technology has been widely used in various products and is well known by people. However, the intelligent face recognition system developed at present lacks universal design concept, and the designed system cannot be applied to various products. During the use of users, there are some problems, such as difficult operation and unfriendly interface. In order to improve the satisfaction of users' physical examination and the accuracy of intelligent face recognition, this study develops an intelligent face recognition system based on the universal design concept. First, the universal design concept is briefly described, and the calculation process of face detection algorithm and face detection algorithm based on the optical flow method is introduced in detail. Then, when designing a face recognition system, this algorithm is used to build a complete system framework. The main functional modules in this system are face detection module, face recognition module, and face training module. The functions of each module are described in detail. Finally, the face feature extraction results of the face detection algorithm based on the optical flow method are verified on the Yale face database and PIE face database. The results show that the algorithm has the highest detection and recognition rate. At the same time, the ORL face database is used to compare and analyze the system performance. The face image recognition rate of this algorithm is 92, which is the highest compared with other algorithms.

## 1. Introduction

As we know that development and innovations in technology are moving on a very fast track, which is due to the fact that various activities in our daily life routine work are required to be automated completely (if feasible and applicable) or partially where these systems are used to assist human beings. These developments are further encouraged with the advent of artificial intelligence such that various tedious and time-consuming task related to the human beings are needed to be carried out through the automated systems, i.e., decision support or management systems. These systems have resolved or in some application areas replaced human beings, especially in those areas where it is hard for an ordinary human being to perform or critical as far as life perspectives of the human beings are considered. These types of automated systems have applications in different research domains such as industries, healthcare, and surveillance system. In these systems, cameras, i.e., both unidirectional and multidirectional, are used to capture timely information about the phenomenon for which it is deployed.

The article "Intelligent Face Recognition System Based on Universal Design Concept" was retracted in 2023. Reasons: signs of a paper mill; suspected computer-generated content; unreliable results or conclusions; concerns about the data.

The emergence of intelligent face recognition technology has changed the interaction mode between human and machine. Now entering the face brushing era, face recognition is widely used in various fields [1]. With the rapid development of science and technology, people's life is more intelligent. More and more people put forward higher requirements for social security prevention and control, hoping to get a more reliable system and improve the universality of face intelligent recognition system. Therefore, this study uses the universal design concept to study the intelligent face recognition system.

The universal design idea is a new design concept that has been offered. The design is more relevant since it is applicable to anybody, independent of human ability, gender, age, or varied settings. To improve the performance of intelligent face recognition and make it universally applicable, an intelligent face recognition system is researched and developed based on the universal design concept that can be used in residential areas, high-end office buildings, shopping malls, banks, and other public places [2].

The main innovations in the research process of this study are as follows: (1) this study briefly outlines the universal design idea, which is also the basic theoretical foundation for the development of intelligent face recognition systems, and then goes into detail about the face detection algorithm, which is the system's core algorithm. (2) The face detection algorithm based on optical flow technique is utilised to extract face features while developing the intelligent face recognition system, and the design of the intelligent face recognition system is finished. Face detection, face identification, and face training are the system's core functional elements [3].

The remainder of the manuscript is organized according to the given items.

In the subsequent section, already available approaches are described in brief where it is mentioned how an approach works and which of the challenging issue is addressed with it. Additionally, we have carried out in what perspectives the approach has limitations. The face recognition algorithm, which is based on the universal technique, is discussed in detail.

The article "Intelligent Face Recognition System Based on Universal Design Concept" was retracted in 2023. Reasons: signs of a paper mill; suspected computer-generated content; unreliable results or conclusions; concerns about the data.

## 2. Related Work

Intelligent face recognition technology was proposed in the 1960s. It has been developed for more than 50 years. With the rapid development of science and technology, this technology has made a major breakthrough and developed a variety of face databases and face recognition algorithms. Meenpal et al. proposed a face recognition algorithm based on principal component analysis (PCA). This algorithm uses different distance measures as matching technology and uses principal component analysis for face feature extraction and data representation. The feature dimension of the generated face image is low [4]. Naji and Hamd believed that different databases and methods should be used to identify people and proposed to use the local binary mode and ternary mode in the texture analysis method for comparative analysis. At the same time, three distance measurement methods, namely, Manhattan distance (MD), Euclidean distance (ED), and cosine distance (CD), were taken into account. After comparative analysis, Ren Lina's recognition rate of Manhattan distance was higher [5]. Okokpujie and John experts pointed out that the face recognition system will be disturbed by factors such as illumination, expression, posture, occlusion, and aging, which will reduce the accuracy of the face recognition system. Here, a face recognition system with fixed illumination is developed by using four-layer neural network (CNN). This system can recognize face images with different degrees of illumination and establish a face recognition system with constant model illumination [6]. Akila et al. put forward a car face recognition system based on biotechnology from the perspective of car safety. Using CV global communication system (GSM) module and Arduino, it provides a low-cost safety system for cars, which can accurately track the position of vehicles [7]. Oualla et al. designed a fast face detection algorithm. Based on the current computing environment, it can comprehensively improve the processing speed of smart frames per second and have higher accuracy [8]. Zhou et al. used convolution in face recognition and detection to preserve image spatial information and highlight the advantages of image processing [9]. Zhang et al. build R-CNN model, use convolutional neural network to extract local features in the image area to complete target detection, abandon the traditional sliding window mode, use image features to predict the size and position of the target to be detected, and modify the position frame regression processing [10]. Li and Yu have developed the latest generation of electronic identification system, which can be used to monitor the suspect in real time, so as to realize the nationwide pursuit [11]. Lu et al. have developed a face recognition technology based on surveillance video, which can identify according to the speed of scanning 36 million pictures per second and then save the image information and classify according to the similarity, which can better track criminals [12]. Ou Yang et al. based on deep learning, a face recognition system is established by organically combining the face detection method, face recognition method, opencv affine transformation method, face attribute recognition, and similarity search method [13].

The article "Intelligent Face Recognition System Based on Universal Design Concept" was retracted in 2023. Reasons: signs of a paper mill; suspected computer-generated content; unreliable results or conclusions; concerns about the data.

## 3. Universal Design Concept and Face Recognition Algorithm

With the advancement in technology, various activities are needed to be carried out through the extensive usage of the automated system, which are based on intelligent technology. Likewise, face recognition is very important, especially in the airport or other secured areas of the countries. To develop and realize these systems, cameras are installed, i.e., fixed and movable, in an area, which is needed to be covered and every camera is connected with a centralized system, where the captured data are fed continuously after a certain time interval. These readings are thoroughly examined through extensive and dedicated procedures to identify potential unwanted persons in the vicinity. In this section, we are going to present the proposed design concept along with a detailed discussion on how this system could possibly resolve the issue.

### 3.1. Universal Design Concept

“Universal design” can also be called omni-directional design. It was first proposed by American Ron mace scholars in the 1980s. The earliest definition is a design that has nothing to do with user gender and gender economic ability and is applicable to all people. The purpose is to use the design to make the product meet the needs of users in terms of usability and aesthetics and will not be affected by personal ability, age, and gender differences, so as to make the designed product more inclusive and adaptable.

The fields covered by universal design mainly include road traffic, product design, packaging design, logo design, etc., which are highly related to people's work and daily life. Universal design uses the “people-oriented” concept to remove all the faults existing during people's use of products, so as to maximize the expansion of product application scope. The core of universal design lies in the design of dynamic things, not in a static state. From the perspective of development and dynamics, it completes the object design and the composition of the system environment, improves its own adjustability, and realizes the adjustment in a certain interval.

The article "Intelligent Face Recognition System Based on Universal Design Concept" was retracted in 2023. Reasons: signs of a paper mill; suspected computer-generated content; unreliable results or conclusions; concerns about the data.

### 3.2. Face Detection Algorithm

The Viola–Jones detector developed in 2011 can improve the detection ability and level in an all-round way. This kind of detection requires the input of face photos, so the camera should collect face images when taking pictures. This restriction limits the actual application range of the algorithm, while the front face is easy to identify systematically and improves the recognition accuracy, so it can be used in the empirical comparison scenarios. The main components of the Viola–Jones algorithm are as follows:

1. Describing faces based on Haar features
2. Acquiring various rectangular features quickly from the integral image
3. Training face features based on ADAPOLST algorithm
4. Building cascade classifier

Aces have a lot in common, such as dimmer light in the eye position than in the face, brighter on both sides of the nose bridge, and darker colour on the lips than surrounding them. The position of a person's brows, eyes, and lips on their face is described by the image's grey level shift. As a result, the face regularity may be defined using the image's grey level change characteristic.

The computation of Haar-like features is a straightforward technique. To cope with the complicated and recurring challenges of Haar-like feature computation, the V–J detector employs a data structure, namely, an integral graph. The formula for calculating integral graphs is as follows:

(1) $$\begin{array}{c} I\left(x,y\right)=\sum x^{\prime }\leq x\sum y^{\prime }\leq yf\left(x^{\prime },y^{\prime }\right). \end{array}$$

The top *I*(*x*, *y*) is the sum of all the pixel points, and *f*(*x*′, *y*′) is the pixel point.

The following formula shows a strong classifier based on AdaBoost:

(2) $$\begin{array}{c} G\left(x\right)=\sin\;g\left(f\left(x\right)\right)\\ =\text{sign}\left(\sum_{m=1}^{m}amGm\left(x\right)\right). \end{array}$$

The following formula shows a weak classifier:

(3) $$\begin{array}{c} Gm\left(x\right):⟶\left\{-1,1\right\}. \end{array}$$

The weak classifier *Gm*(*x*) coefficients are calculated from the following formula:

(4) $$\begin{array}{c} a_{m}=\frac{1}{2}\log\frac{1-e_{m}}{e_{m}}. \end{array}$$

Classification errors in formulas are expressed by *e*_*m*_.

In universal, a large number of strong classifiers need to be trained, and multiple strong classifiers need to be cascaded to improve performance. As a result, the input size of the strong classifier can be reduced, the redundant information in the background can be fully considered, and the overall consumption time can be reduced. In addition, the joint enhancement classifier can improve the accuracy of the check.  Figure 1 shows the cascade classifier detection process for face detection:

The article "Intelligent Face Recognition System Based on Universal Design Concept" was retracted in 2023. Reasons: signs of a paper mill; suspected computer-generated content; unreliable results or conclusions; concerns about the data.

### 3.3. Face Detection Based on the Optical Flow Method

The optical concept was first introduced in the 1950s. The optical field is a motion field formed by mapping on a two-dimensional image. The optical flow field can accurately calculate the relative moving vectors of each pixel point and the previous frame in an image sequence. The concept is that if T-frame (*x*_1_, *y*_1_) represents the position of A, then *t*+1 looks for A again, and its position is represented by (*x*_2_, *y*_2_), and point A motion can be obtained by using the following formula:

(5) $$\begin{array}{c} \left(u_{1},v_{1}\right)=\left(x_{2},y_{2}\right)-\left(x_{1},y_{1}\right). \end{array}$$

Face is a three-dimensional structure, and its motion generates images that are different from video motion and two-dimensional planar photographs. Especially in a rotating environment, a variety of optical flow calculation methods are selected. The goal is the same; that is, each pixel requires a corresponding *S* position vector and covers the location information of the pixel movement, as follows:

(6) $$\begin{array}{c} S=\left(\frac{d_{x}}{\overset{⟶}{x}},\frac{d_{y}}{\overset{⟶}{y}}\right)\\ =\left(v_{x},v_{y}\right). \end{array}$$

The optical flow is calculated using the Farneback procedure in this case. The goal of computing the optical flow is to determine whether the identical spatial location will appear in the future frame. To smooth the optical flow field findings, the input colour image should be treated with Gaussian blur first when inputting the image, which is compatible with the premise that the change of vector field is essentially smooth.

Assuming that an image is a two-dimensional signal function, then the dependent variable is the two-dimensional coordinate position *x*=(*x*, *y*)^*T*^, and the image model can be approximately established by using two-dimensional polynomials to obtain the following results:

(7) $$\begin{array}{c} f\left(x\right)∼X^{T}AX+b^{T}X+C. \end{array}$$

The above *b* is the vector, *A* is the symmetric matrix, and the image model is as follows:

(8) $$\begin{array}{c} f_{1}\left(x\right)=X^{T}A_{1}X+b_{1}^{T}X+c_{1}. \end{array}$$

The image of the second frame *f*_2_(*x*) after the pixel offset is as follows:

(9) $$\begin{array}{c} f_{2}\left(x\right)=f_{2}\left(x-d\right)\\ ={\left(X-d\right)}^{T}A_{1}\left(X-d\right)+b_{1}^{T}\left(X-d\right)+c1⟶f_{2}\left(x\right)\\ =X^{T}A_{1}X+{\left(b_{1}-2A_{1}d\right)}^{T}A+d^{T}A_{1}d-b_{1}^{T}+c_{1}⟶f_{2}\left(x\right)=X^{T}A_{2}X+b_{2}^{T}X+c_{2}. \end{array}$$

The above formula has the following relationship:

(10) $$\begin{array}{c} \left\{\begin{array}{c} A_{2}=A_{1},\\ b_{2}=b_{1}-2A_{1}d,\\ c_{1}=d^{T}A_{1}d-b_{1}^{T}+c_{1}. \end{array}\right. \end{array}$$

On substituting formula (10) in the following formula, we obtain

(11) $$\begin{array}{c} 2A_{1}d=-\left(b_{2}-b_{1}\right)⟶d\\ =-\frac{1}{2}A_{1}^{-1}\left(b_{2}-b_{1}\right). \end{array}$$

An initial displacement exists at each pixel point, and by adding the initial displacement of the previous frame to the x-pixel point, the local pixel position $\tilde{x}$ on the next frame of the image can be obtained. $\tilde{x}=x+\tilde{d}\left(x\right)$, where $\tilde{x}$ is a floating point location and it is difficult to predict the coefficient vector values at this location. This study deals with this problem by rounding the initial displacement to obtain an integer and using it in the intermediate variables *A*(*x*) and Δ*b*(*x*). The following relationships exist:

(12) $$\begin{array}{c} A\left(x\right)=\frac{A_{1}\left(x\right)+A_{2}\left(x\right)}{2},\\ A\left(x\right)d\left(x\right)=\Delta b\left(x\right),\\ \Delta b\left(x\right)=-\frac{1}{2}\left(b_{2}\left(x\right)-b_{1}\left(x\right)\right). \end{array}$$

*S*(*x*) is a scale matrix, *h*(*x*) is an intermediate variable, and *G*(*x*) is calculated as follows:

(13) $$\begin{array}{c} G\left(x\right)=S{\left(x\right)}^{T}A{\left(x\right)}^{T}A\left(x\right)S\left(x\right),\\ h\left(x\right)=S{\left(x\right)}^{T}A{\left(x\right)}^{T}\Delta b\left(x\right). \end{array}$$

Based on the precondition that most of the photorheological changes are smooth, the optical flow field is calculated after fuzzification of *G*(*x*) and *h*(*x*):

(14) $$\begin{array}{c} d_{\text{out}}\left(x\right)=G_{\text{avg}}{\left(x\right)}^{T-1}h_{\text{avg}}\left(x\right). \end{array}$$

This vector involves the size and direction of the pixel point displacement. The number of motion is decomposed to *X*-axis and *Y*-axis. After normalization, a value interval of 0–255 can be used.  Figure 2 shows the overall architecture of this algorithm.

The article "Intelligent Face Recognition System Based on Universal Design Concept" was retracted in 2023. Reasons: signs of a paper mill; suspected computer-generated content; unreliable results or conclusions; concerns about the data.

## 4. Intelligent Face Recognition System Based on Universal Design Concept

Intelligent or smart system, which is specifically developed for the recognition of face, is presented here in detail. It is important to note that this system should incorporate the required level of the intelligence, which are needed to improve accuracy and precision ratio of the system. For this purpose, various cameras have been deployed in the closed proximity of the individual, which are needed to be identified. For this purpose, these cameras are installed in locations where it is highly likely that each and every individual is seen and his images are captured.

### 4.1. Design of the Face Recognition System

This study establishes a face recognition system based on the universal design concept, which is used for static face image recognition [14]. In practical application, it is necessary to use the combination of multifeature detection to segment and detect faces. After that, the feature vectors on the face are extracted using the PCA-based feature extraction algorithm, and the Euclidean distance criteria are used for identity matching. In this study, Euclidean distance is selected to identify features. Since the complexity of this method does not affect the real-time performance of the system, the face recognition results will be output after the end.  Figure 3 shows a system flowchart.

Figure 3 shows the system design framework, with the dashed line frame representing the system's algorithm. In the dashed line frame below, the primary method of facial recognition [15] is listed. The system is made up of a data processing module, a foreground human-computer interface module that is used to pick the input picture source, face recognition, and the output of face recognition results. Face detection, face recognition, and face feature extraction are the core modules of this approach.

### 4.2. System Module Design

Figure 4 shows the system module design framework.

The main modules in the running process of the face recognition system designed and developed in this study are the registration login module, image acquisition module, face detection module, face recognition module, face training module, wireless communication module, and wired communication module [16]. At the same time, a high-definition camera is installed on the desktop computer with the system as Windows l0, and Stable Build WeChat developer tools, CSS cascading style sheets, HTML markup language, and JavaScript scripting language are used to design and implement the system home page, face registration page, face detection page, and face recognition page through programming. There are a fast-running development framework, a large number of components, and APIs in the WeChat developer tools to assist developers in providing an APP service experience using the development tools. Face registration, face detection, and face login pages all call the camera API implementation on the WeChat applet to call the camera function and photo-taking function. By combining with a timer, setting an interval of 50 ms to call the camera API interface to complete the photo-taking operation, and realizing the function of timer photo taking, we can get the real-time picture in this camera [17].

The article "Intelligent Face Recognition System Based on Universal Design Concept" was retracted in 2023. Reasons: signs of a paper mill; suspected computer-generated content; unreliable results or conclusions; concerns about the data.

The process of designing and implementing each function page on the client is as follows:

1. *Face Registration Page, Face Detection Page, and Face Login Page*. We should complete the regular opening and jumping of three pages while developing the home page, face registration page, face detection page, and face login page.
2. Two buttons, face recognition, and face detection are established while constructing the system's main page. After pressing the face detection function, the user may navigate to this page and utilise the back-end service to access the image upload interface and the face detection module interface. The associated menu bar will open up from the bottom after activating the facial recognition function, allowing you to pick the correct menu bar. The functions shown on the menu bar are the face registration, login, and cancel buttons. After pressing this function, it will automatically jump to the face registration interface [18]. Pressing the login function will jump to the login interface, and clicking cancel will close the menu bar and go to the home page.
3. *Face Detection Interface*. The purpose of this interface is to monitor a face picture in real time in a window and finish the drawing of a face frame in the page display window. To perform the face detection function, the top left corner and lower right corner of the face frame will be presented on the information frame with the vertical coordinates.
4. After pressing the start button, the client will automatically call the timer and camera API interface, take pictures every 50 milliseconds, then upload the picture information to the back-end server side, upload the image to the service side, and make additional calls to the face detection module interface to complete face detection and return face frame coordinate information to the client. The feedback face frame coordinate data are parsed on the client side, and the face frame drawing operation is completed in the display window. Finally, in the information frame, the upper left corner and lower right corner of my face frame are output in the horizontal and vertical coordinate values. The stop button is pressed to pause face detection.
5. *Face Registration Interface*. This interface is achieved by taking pictures of the page to display the screen in the window and completing face feature extraction, the extracted face features will be displayed in the window, and the face registration operation will finish when the information is written in the database.
6. After pressing the face acquisition function, the client must call the camera API function to complete the photo-taking operation, after which the registered picture can be obtained, the image upload interface on the background server can be called, the collected image information can be transferred to the server, the face registration module interface can be called to realize face detection and face feature extraction, and the detected coordinate information of the detected face can be obtained. The collected coordinate information of the face frame is parsed on the client side, the display window completes the face frame's location, and the interface shows the “acquisition success” reminder after completion. If the registered image is not approved, we can delete all the collected forehead face images by pressing the empty function, then tap the face collection function to recollect the face feature information according to the above process, complete the face registration, and fill in the face image information in the corresponding registration information table of the database.
7. *Face Logon Interface*. This function detects the screen on the display window, extracts the face feature values from the screen, calculates the Euclidean distance between the feature values and the registrant's face feature values, determines whether the logon and the registrant are consistent based on the Euclidean distance, and ends the face recognition operation.

The article "Intelligent Face Recognition System Based on Universal Design Concept" was retracted in 2023. Reasons: signs of a paper mill; suspected computer-generated content; unreliable results or conclusions; concerns about the data.

## 5. Analysis of Face Recognition Results

This section discusses an extensive summary of the observation, which is perceived during the evaluation process of the proposed and existing systems is reported. Initially, results related to the recognition of face are presented.

### 5.1. Analysis of Face Recognition Results

This study establishes an intelligent face recognition system based on the universal design concept and selects the Yale face database and PIE face database to judge and analyze the face recognition effect of this system [19]. By using the face detection algorithm based on optical flow to complete the face feature extraction, we use the European classifier to judge the face image can improve the face recognition effect. The results of face recognition in Yale and PIE face databases by ANMM are compared with those obtained by this algorithm. The results are shown in Figures 5 and 6.

The face identification algorithm based on optical flow approach utilised in this study is more separable than the ANMM algorithm, according to the results provided in Figures 5 and 6. Traditionally, the issue must be divided before the trajectory can be calculated. This approach is straightforward; however, it lowers computation accuracy. When computing the W-feature mapping issue in this study, the optical flow face identification method conducts a division operation after tracing and then solves it using an iterative approach. Compared to the old technique, this algorithm's W-feature mapping matrix may collect smaller data points of the same kind while pushing away data points of different types.

The article "Intelligent Face Recognition System Based on Universal Design Concept" was retracted in 2023. Reasons: signs of a paper mill; suspected computer-generated content; unreliable results or conclusions; concerns about the data.

This study chooses several algorithms to compare the recognition rate of each algorithm, such as the PCA algorithm, PCA + LDA algorithm, ANMM algorithm, and this algorithm. Comparing the face recognition rate of these algorithms on Yale and PIE face databases, the results obtained are listed in Table 1.

Analyzing the results obtained in Table 1, it is shown that the recognition rate obtained by this algorithm on the PIE face database is significantly higher than that of Yale face database, and the face detection algorithm based on the optical flow method used in this study has the highest recognition rate. The factors leading to this result are that the recognition rate varies greatly in different databases due to illumination, face angle, and other factors.

### 5.2. System Performance Analysis

In this study, we validate the intelligent face recognition system based on the universal design concept and analyze the performance with the ORL face database combined with the face recognition test scheme, which is used to judge the performance of face recognition in life and in standard face database [20]. When testing the face recognition performance of this system on a standard face database, the ORL face database face image is selected as the test object, and the results are listed in Table 2. Each person in the face database has 10 face images, and 10 persons are selected, so the total image number will be 100. Each face image has a certain difference in shooting angle, time, facial decorations, facial expressions, etc. Another 10 face images used are 5 females and 5 males. There are images taken and collected systematically in the images to be recognized, including personal travel photos or certificate photos. The selected light, shooting angle, and expression of the certificate photos are basically unchanged.  Figure 7 shows face recognition speed and recognition rate results.

Combined with the data in Table 2 and Figure 7, the face recognition system designed in this study basically meets the expected requirements and has a strong real-time face recognition and highest recognition rate. The system can recognize 92% of the face images in ORL face database, and the recognition accuracy is over 80% when recognizing life photos and standard photos, and the recognition speed and recognition rate of standard face database are higher than those of self-built face database. This demonstrates that during face identification, facial expression, ambient illumination, a backdrop with a strong resemblance to skin tone, and the shooting angle all impact the face recognition rate. Because standard illuminations are mostly colourful, it takes a long period of time to process as there are a large amount of hidden information. The speed of recognition standard illumination is lower than that of the face database, but its recognition efficiency is higher than that of the ORL face database.

The article "Intelligent Face Recognition System Based on Universal Design Concept" was retracted in 2023. Reasons: signs of a paper mill; suspected computer-generated content; unreliable results or conclusions; concerns about the data.

## 6. Conclusion

The rapid development of science and technology has gradually entered people's lives. With the increase of storage capacity and computing speed on hardware, more products about face recognition have been initially developed, which will change the interaction mode between people and computers. Face recognition technology, which uses noncontact and visualization features, has been widely used in security, payment, and other fields. However, the face recognition system developed is not universal and cannot be used in various fields. For this problem, this study uses the universal design concept to develop an intelligent face recognition system, breaking the barriers that traditional systems cannot be applied in other areas, to achieve comprehensive promotion and use and improve the efficiency of face recognition. By describing the universal design concept and face detection algorithm in detail, an intelligent face recognition system based on the universal design concept is built, and the face recognition operation is completed with the system. This study chooses the ORL face database to test the system performance. The result shows that the face recognition rate of this system is 92%, which is the highest compared with other algorithms.

## Figures and Tables

**Figure 1:** Face detection process.

**Figure 2:** Overall architecture of optical flow face detection.

**Figure 3:** System flowchart.

**Figure 4:** System module framework.

**Figure 5:** Comparison of recognition results of Yale face database.

**Figure 6:** Comparison of recognition results for PIE face database.

**Figure 7:** Line chart of system test results.

**Table 1:** Comparison of recognition rates of different algorithms.

	PCA (%)	PCA + LDA (%)	ANMM (%)	This algorithm (%)
Yale face database	57.4	72.6	72.9	75
PIE face database	54.5	87.1	93.2	96.1

**Table 2:** System test results.

Project	Total faces	Number of errors	Recognition rate (%)	Recognition speed (MS)
ORL face database	100	8	92	336
Life photos	50	10	80	635
Standard photo	50	3	94	458

The article "Intelligent Face Recognition System Based on Universal Design Concept" was retracted in 2023. Reasons: signs of a paper mill; suspected computer-generated content; unreliable results or conclusions; concerns about the data.

## Data Availability

The datasets used and/or analyzed during the current study are available from the corresponding author upon reasonable request.
